# Enhancing Disease Classification in Abdominal CT Scans through RGB Superposition Methods and 2D Convolutional Neural Networks: A Study of Appendicitis and Diverticulitis

**DOI:** 10.1155/2023/7714483

**Published:** 2023-05-29

**Authors:** Gi Pyo Lee, So Hyun Park, Young Jae Kim, Jun-Won Chung, Kwang Gi Kim

**Affiliations:** ^1^Department of Health Sciences and Technology, Gachon Advanced Institute for Health Sciences and Technology (GAIHST), Gachon University, Incheon, Republic of Korea; ^2^Department of Radiology, Gil Medical Center, Gachon University College of Medicine, Incheon, Republic of Korea; ^3^Department of Biomedical Engineering, College of IT Convergence, Gachon University, Gyeonggi-do, Republic of Korea; ^4^Division of Gastroenterology, Department of Internal Medicine, Gil Medical Center, Gachon University College of Medicine, Incheon, Republic of Korea; ^5^Department of Biomedical Engineering Medical Center, College of Medicine, Gachon University, Incheon, Republic of Korea

## Abstract

The primary symptom of both appendicitis and diverticulitis is a pain in the right lower abdomen; it is almost impossible to diagnose these conditions through symptoms alone. However, there will be misdiagnoses happening when using abdominal computed tomography (CT) scans. Most previous studies have used a 3D convolutional neural network (CNN) suitable for processing sequences of images. However, 3D CNN models can be difficult to implement in typical computing systems because they require large amounts of data, GPU memory, and extensive training times. We propose a deep learning method, utilizing red, green, and blue (RGB) channel superposition images reconstructed from three slices of sequence images. Using the RGB superposition image as the input image of the model, the average accuracy was shown as 90.98% in EfficietNetB0, 91.27% in EfficietNetB2, and 91.98% in EfficietNetB4. The AUC score using the RGB superposition image was higher than the original image of the single channel for EfficientNetB4 (0.967 vs. 0.959, *p* = 0.0087). The comparison in performance between the model architectures using the RGB superposition method showed the highest learning performance in the EfficientNetB4 model among all indicators; accuracy was 91.98% and recall was 95.35%. EfficientNetB4 using the RGB superposition method had a 0.011 (*p* value = 0.0001) AUC score higher than EfficientNetB0 using the same method. The superposition of sequential slice images in CT scans was used to enhance the distinction in features like shape, size of the target, and spatial information used to classify disease. The proposed method has fewer constraints than the 3D CNN method and is suitable for an environment using 2D CNN; thus, we can achieve performance improvement with limited resources.

## 1. Introduction

The primary symptom of both appendicitis and diverticulitis is a pain in the right lower abdomen; diagnosis of these diseases using symptoms alone is nearly impossible. Diagnosis is performed using abdominal computed tomography (CT); abdominal ultrasound examination or magnetic resonance imaging (MRI) can also be used depending on the situation [1–4]. However, it is known that over 70% of diverticulitis patients undergo surgery owing to an initial diagnosis of appendicitis [5, 6]. The rate of missed diagnosis of appendicitis in emergency department visits is 3.8-15% in children and 5.9-23.5% in adults, which can be especially confounding when patients present with atypical symptoms [7]. And according to Lee and Hyun [8], 80% of patients with diverticulitis had been misdiagnosed as having appendicitis initially (before surgery).

Several studies have been conducted to classify appendicitis and diverticulitis using artificial intelligence techniques such as machine learning or deep learning to overcome the aforementioned difficulties. Marcinkevics et al. and Pati et al. [9, 10] developed predictive models for appendicitis diagnosis using several machine learning algorithms like logistic regression, random forests (RF), and gradient boosting machines to predict on 430 children and adolescents aged 0 to 18. They showed an accuracy of 91.57% and a sensitivity of 91.95% on the appendicitis diagnosis model using RF. And using ensemble-learning techniques on the majority voting ensemble classifiers, they obtained an accuracy of 92.15% and a sensitivity of 95.02%. Park et al. investigated a neural network-based diagnosis algorithm for diagnosing appendicitis by using CT. They trained a three-dimensional convolutional neural network (3D CNN) for use in binary classification that distinguishes between an appendix with appendicitis and a normal appendix, using 3D CT data. The results exhibited an accuracy of 0.915, and the sensitivity and specificity values were 0.902 and 0.920, respectively [11]. Rajpurkar et al. developed a model called AppendiXNet to detect appendicitis. AppendiXNet used a 3D residual network (3D ResNet) architecture and was pretrained on a large dataset called “Kinetics.” Performance evaluation of AppendiXNet revealed an area under the curve (AUC) of 0.810, a sensitivity of 0.667, and a specificity of 0.784 on the test dataset [12].

Most studies for the classification of appendicitis and diverticulitis use 3D CNN models suitable for processing sequences of images. Unlike a 2D CNN that learns using 2D feature information, a 3D CNN extracts 3D feature information, including spatial data, and uses it for deep learning. The coronal or sagittal image generated through a 3D reconstruction of the abdominal CT image is used to determine the location or presence of appendicitis and diverticulitis. When diagnosing appendicitis and diverticulitis in the clinic, judgment is not based on a single image; a complex assessment is performed by referring to the previous and next slices of the corresponding images. Therefore, even for deep learning training, using continuous images for prediction is more effective than using a single image.

Despite the aforementioned advantages, there are many constraints in using 3D CNNs. 3D CNN models used in deep learning require substantially more training data than 2D CNN models. However, it is difficult to collect large amounts of medical data, such as CT and MRI data, for reasons like being strictly regulated for privacy and security and the difficulty of sharing datasets with other researchers [13, 14]. In addition, there are few 3D CNN models pretrained using large datasets to utilize transfer learning; this presents challenges in deep learning. Moreover, the architecture of 3D CNN models is required to process a large amount of data information and perform complex computational processing, which demands high-end hardware specifications and takes a considerable amount of time [15].

In this study, we propose a deep learning method by applying an RGB channel superposition image reconstructed from three slices of sequence images in CT data to 2D CNN models, which enables learning like 3D CNN models. We evaluated the performance of the proposed deep learning method by comparing the training results obtained using the original image with those obtained using the RGB superposition image. In addition, to confirm the advantage of using more feature information from the image, we trained and evaluated several models having different numbers of parameters and compared their performance.

## 2. Materials and Methods

### 2.1. Data

In this study, to verify the effectiveness of deep learning using RGB superposition images, we collected abdominal CT images of a total of 500 patients (male : female, 265 : 235; mean age ± standard deviation, 43.35 years ± 16.63) including 246 patients (male : female, 128 : 118; mean age ± standard deviation, 42.02 years ± 19.16) with appendicitis and 254 patients (male : female, 137 : 117; mean age ± standard deviation, 44.65 years ± 13.65) with diverticulitis from CT scans performed at the Gil Medical Center from January 2017 to January 2020. This data collection was approved by the institutional review board (GAIRB2020-096) of Gachon University Gil Hospital. The requirement for informed consent was waived according to the ethical standards of the institutional review board.

CT images were taken by CT scanners including SOMATOM Edge, SOMATOM Definition AS, SOMATOM Definition Flash, and SOMATOM Force (Siemens Healthcare). The scan parameters of the CT scanner were tube voltages of 80, 100, or 120 kVp and varied reference tube currents of 170–298 mAs. The dimensions of the CT images were 512 × 512, and the pixel spacing ranged between 0.46 and 0.97 mm/px; the slice thickness was 3–5 mm.

From the abdominal CT images collected, 2,782 axial-slice images were used: 1,959 images of patients with appendicitis and 823 images of patients with diverticulitis. The images of appendicitis and diverticulitis were annotated, including the surrounding region of inflammation. Using the ImageJ software (NIH, Bethesda, MD, USA), experts manually annotated appendicitis and diverticulitis regions in the collected axial CT images through box-type annotations.

### 2.2. RGB Superposition Image

We cropped the box-shaped regions of interests (ROIs) from the start to the end position of appendicitis and diverticulitis based on an expert's manual annotation. Additionally, to generate RGB superposition images, we extracted images of the previous and next slices from the positions of the first and last disease areas. The cropped images were resized to the input shapes expected for each EfficientNetB0, B2, and B4 base model (resolution: 224 × 224, 260 × 260, and 380 × 380).

We resized the extracted previous and next slice images to the size of the ROI image. Then, we converted the ROI image to a color image with three channels: red, green, and blue channels. Replacing the red and blue channels of the ROI image with the previous and next slice CT images, respectively, we obtained an RGB superposition image including three image slices. This process is depicted in Figure 1. The RGB superposition images were used to train and test data for deep learning training. Some samples of RGB superposition images of appendicitis and diverticulitis are presented in Figure 2.

We obtained 1,959 original images of appendicitis and 823 original images of diverticulitis from the CT images of the 500 patients, and the corresponding number of RGB superposition images was generated for each disease. The number of images of diverticulitis was insufficient compared to the number of appendicitis images; the imbalance of training data could have resulted in poor performance and overfitting of the classification training. To prevent this, the number of images of diverticulitis was brought to a value close to the number of appendicitis images through data augmentation. We applied image-processing methods such as rotation, width shift, height shift, and zoom and varied the hyperparameters randomly across specified ranges to generate fake diverticulitis images. We added the generated fake diverticulitis image to the training dataset and applied it to the training models.

### 2.3. Experimental Environment

The system for deep learning employed IBM Power System AC922 8335-GTH (IBM, Armonk, NY, USA) with a single NVIDIA Tesla V100-SXM2 16GB (NVIDIA, Santa Clara, CA, USA). The operating system used was Ubuntu 18.04.3. We used Python (version 3.7.11) with TensorFlow frameworks (version 2.2.0) for training and testing deep learning networks. For image processing, the OpenCV-python 4.1.1, Pydicom 2.2.2, and read-roi 1.6.0 libraries were used.

### 2.4. Deep Learning

To verify performance enhancement using the RGB superposition images for deep learning, this study compared the performance of several training models using the original images and the RGB superposition images. Deep learning training to classify appendicitis and diverticulitis was conducted to evaluate the model's performance. The flowchart in Figure 3 depicts the deep learning process used in this study.

The original and RGB superposition images were trained and tested using EfficientNetB0, B2, and B4 models pretrained on ImageNet by transfer learning. Transfer learning is a technique for deep learning that uses pretrained neural network weights as a starting point for large and diverse datasets such as ImageNet. This is a popular way to shorten the model's learning time and computational resources and improve the model's performance on a small image dataset because the features learned by the pretrained model can be applied to a new task regardless of the subject with little modification. The input data was resized to corresponding dimensions of 224 × 224, 260 × 260, and 380 × 380 to use transfer learning for each model, respectively. The hyper-parameters of training used were as follows: the number of epochs was 200; the batch size was 64; and the base learning rate was 0.0001 (le-4) and decreased to 0.00001 (le-5) when the number of epochs was greater than 30. We adapted that the training process stopped when validation loss has not improved during the 10 epochs to void overfitting.

### 2.5. Performance Evaluation

In this study, the performance of deep learning methods using the original and RGB superimposition images was compared through the classification of appendicitis and diverticulitis. Model performance was evaluated by performing 5-fold cross-validation. Cross-validation is a technique used to assess the reliable estimation performance of a training model and how the model will perform on unseen data. This process typically involved splitting the training dataset into *k* subsets of roughly equal size and calling each subset like “fold,” in this study, we divided 5 folds. The model is then used a fold as for testing performance and trained to the remaining folds (*k* − 1 folds). This process is repeated *k* times, with different folds being used as the test set each time. The performance of the model on the *k* test sets is then averaged to produce a final single performance metric [16]. Each fold was configured by dividing the number of images similarly, based on the patient, to prevent overfitting. The trained prediction model's performance was evaluated on the basis of accuracy, precision, and recall [17]. Additionally, the receiver operating characteristic (ROC) curve and area under the curve (AUC) scores were utilized for the assessment. The ROC analysis and comparison were performed using MedCalc version 19.6.1 for Windows (MedCalc Software, Ostend, Belgium).

## 3. Results

In this study, we trained and tested models for the classification of appendicitis and diverticulitis. Through 5-fold cross-validation, all the data were used for model validation, and the confusion matrix determined using the model was synthesized to form the confusion matrix for all the data. In the confusion matrix for appendicitis and diverticulitis classification, true positive (TP) was a case that classified appendicitis as appendicitis, false negative (FN) was a case that classified appendicitis as diverticulitis, false positive (FP) was a case that classified diverticulitis as appendicitis, and true negative (TN) was a case that classified diverticulitis as diverticulitis.

Statistical measures of the performance, such as accuracy, precision, and recall, were calculated; the resulting values are presented in Table 1. Overall, the models that used the RGB superposition images as input images outperformed those that were inputted with original images. In particular, using the RGB superposition image improved accuracy by 2.23% and 2.33% (each EfficientNetB0 and EfficientNetB4) and recall by 1.27%, 1.48%, and 3.26% (each EfficientNetB0, EfficientNetB2, and EfficientNetB4). The AUC scores and comparison results are presented in Table 1, and the ROC curves are shown in Figure 4. The AUC score using RGB superposition images were higher than those with original images for EfficientNetB0 (0.956 vs. 0.948, *p* = 0.0133), EfficientNetB2 (0.962 vs. 0.955, *p* = 0.0246), and EfficientNetB4 (0.967 vs. 0.959, *p* = 0.0087). Among three models that used RGB superposition images, EfficientNetB4 model exhibited the highest training performance with an accuracy of 91.98 (vs. 90.98, 91.27) and recall of 95.35 (vs. 94.38, 95.25). EfficientNetB4 had a 0.011 AUC score higher than EfficientNetB0, and the *p* value was 0.0001, showing a significant difference.  Figure 5 shows grad-class activation map (Grad-CAM) [18] images of the prediction of EfficientNetB0 models. In the case of using the RGB superposition image, the distribution of the red color on the heat map that indicates higher importance for predicting the class correctly was focused more on the center location of appendicitis and diverticulitis.

## 4. Discussion

In this work, we compared the performance of the trained prediction models for the classification of appendicitis and diverticulitis, for the cases wherein the original image was generated from one CT slice image and those wherein the RGB superposition image was generated using three consecutive CT slice images. The proposed method using the RGB superposition images demonstrated better performance, improving the accuracy by 2.23%, 2.33%, precision by 1.8%, 0.27% in EfficientNetB0 and B4, and recall (sensitivity) by 1.48%, 3.26% in EfficientNetB2 and B4 compared to the method using the original images. The AUC score was 0.956, 0.962, and 0.967 in EfficientNetB0, B2, and B4, respectively; all AUC scores of methods using RGB superposition image were higher than methods using single image (0.948, 0.955, and 0.959), and the *p* value was 0.0133, 0.0246, and 0.0087, confirming that our method was statistically significant (*p* < 0.05). The results of the experiment suggested that the classification performance using this method was higher than that using commonly used training methods, which use single images in 2D CNN models.

When the number of parameters of the model is increased, more feature information has the advantage of obtaining more higher performance and preventing overfitting [19, 20]. Each model's total parameters were 4,052,126 in EfficientNetB0, 7,771,380 in EfficientNetB2, and 17,677,402 in EffcientNetB4. EfficientNetB4 which had the highest number of parameters showed the highest performance in all indicators. In CNN models, it was seen that there is a major correlation between accuracy improvement and model size; accuracy increased as the size of the model increased. However, the increase in the number of model parameters led to an increase in computational quantity and training time. In this study, the average number of epochs at the moment of the occurrence of the early stopping was lower when RGB superposition images were used as input images (47.6 epochs) compared to the original images (53.2 epochs) in EfficientNetB4. Additionally, the comparison among the models using the RGB superposition method revealed that the model returned the highest performance with the shortest training time, as the occurrence of early stopping was at 47.6 epochs, compared to 50.4 epochs in EfficientNetB2 and 126.6 epochs in EfficientNetB0. The results show that as the number of model parameters and the amount of computational quantity increases, the RGB superposition method effectively utilized more feature information to show high performance for a short time. The Grad-CAM was generated to visualize the specific class image as a heat map. It provides the location information where the CNN model has focused when predicting a specific class image as the correct class by highlighting the important area. In the case of a model using the RGB superposition method, it can be seen that the center of the heat map appears in the inflammatory region compared to the case using the original method. This indicates that the learning model succeeded in classifying with a weight on the inflammatory site in the process of classifying.

## 5. Conclusion

In almost all cases, 3D CNN provides superior performance than 2D CNN because more information is used in combination [21]. However, using 3D CNN is relatively challenging, depending on the characteristics or the number of data; it demands more computational resources and high-end hardware performance for training [17, 22]. The method proposed in this study presents fewer constraints than methods using 3D CNN and is suitable for an environment using 2D CNN; therefore, it can easily achieve performance improvement in an environment with limited resources. Especially, the proposed method will be useful for the segmentation of whole organs as well as a classification to determine disease presence when 3D medical images such as CT and MRI are utilized for 2D CNN.

An RGB superposition image refers to a fake image with the image information of the previous and next slices of the image combined together and used for prediction. In this study, using the RGB superposition image, the continuous relationship between the previous and next CT slice images was utilized in the process of extracting the feature map from the convolutional layers in the model training process. The training process was enhanced by using more feature information than the traditional 2D CNN models, which use only a single slice image. The superposition of sequence images is applied to enhance the distinction in features used to classify disease. The primary difference between appendicitis and diverticulitis is the disease position. The sequential image information in an RGB superposition image can help in assessing the feature information of the position where the disease occurs. In addition, information such as the continuous shape of the appendix or colon diverticulum and the location or size of the inflamed area is valuable for classification in deep learning training.

This study proposed a deep learning training method which is called the RGB superposition method based on 2D CNN using RGB superposition images. We developed and compared performance for 2D CNN models using EfficientNetB0, B2, and B4 architectures to classify appendicitis and diverticulitis on single and RGB superposition images. The RGB superposition method showed higher performance than the traditional method. And as the model's layers were more used and deeper, training performance was better. These showed more feature information from the sequential images for RGB superposition images worked effectively on the training progress of the deep learning model.

Our proposed method had some limitations. (1) We compared the results of deep learning training with RGB superposition images and original images to confirm that the proposed method performs better on 2D CNN, but we failed to proceed with the comparison with 3D CNN and RGB superposition images. (2) We collected and developed the CNN models using an image, which was collected from some predefined patient cases; we lack variety and need more generality in the model. We would collect more data including normal patients' CT images and various patients' cases in the future; performance and generality can be expected to be improved through retraining. Furthermore, we will confirm the effectiveness of our proposed method through a comparison between 2D CNN model performance using RGB superposition images and the performance of 3D CNN models like 3D-ResNets. We would develop a computer-aided diagnosis (CAD) that can be utilized in emergency rooms, and radiology by developing optimized models through the development of image preprocessing algorithms, model architecture, and hyperparameter coordination. And, for using CAD in practice, a study would be needed to develop an automatic detection algorithm for appendicitis or diverticulitis region.

## Figures and Tables

**Figure 1:** Process of generating RGB superposition images.

**Figure 2:** Sample images of RGB superposition method: (a) appendicitis, (b) diverticulitis.

**Figure 3:** Process flowchart comparing the performance of training models using the original images and RGB superposition images.

**Figure 4:** Comparison of the ROC curves of each model trained from the two different methods for input data (evaluated on the test data according to cross-validation). For all models, the model using RGB superimposed images showed higher prediction performance (as AUC closer to 1 indicates higher performance), and using EfficientNetB4 showed the best performance than other architecture: (a) EfficientNetB0; (b) EfiicientNetB2; (c) EfficientNetB4.

**Figure 5:** Samples of Grad-CAM overlaid on images correctly classified by the EfficientNetB0 model. The activation area for the model's prediction using RGB superposition images showed a more accurate representation of the inflamed area than using the original images.

**Table 1:** The accuracy, precision, recall, and AUC of the final model are calculated by averaging over the performance of the test sets according to cross-validation.

Model name	Accuracy, % (95% CI)	Precision, % (95% CI)	Recall, % (95% CI)	AUC (95% CI)	*p* value^∗^
Original image					
EfficientNetB0	88.75 (87.52-89.90)	91.11 (89.90-92.11)	93.11 (91.90-94.19)	0.948 (0.939-0.956)	
EfficientNetB2	90.47 (89.32-91.54)	92.78 (91.71-93.72)	93.77 (92.61-94.80)	0.955 (0.946-0.962)	
EfficientNetB4	89.65 (88.46-90.76)	93.13 (92.07-94.07)	92.09 (90.80-93.24)	0.959 (0.951-0.966)	
RGB superposition image					
EfficientNetB0	90.98 (89.85-92.02)	92.91 (91.86-93.84)	94.38 (93.27-95.36)	0.956 (0.948-0.964)	0.013
EfficientNetB2	91.27 (90.15-92.29)	92.56 (91.50-93.50)	95.25 (94.22-96.15)	0.962 (0.954-0.969)	0.025
EfficientNetB4	91.98 (90.91-92.97)	93.40 (92.37-94.30)	95.35 (94.33-96.24)	0.967 (0.960-0.974)	0.009

^∗^ *p* value was compared with between results of the two different methods using the same model architecture.

## Data Availability

The datasets used to support the findings of this study are available from the corresponding author upon request.
